This article has been retracted.

# Network Pharmacology and Molecular Docking-Based Investigation of Potential Targets of Astragalus membranaceus and Angelica sinensis Compound Acting on Spinal Cord Injury

**DOI:** 10.1155/2022/2141882

**Published:** 2022-09-15

**Authors:** Shengnan Cao, Guangjian Hou, Ya Meng, Yuanzhen Chen, Liangyu Xie, Bin Shi

**Affiliations:** ^1^School of Acupuncture and Tuina, Shandong University of Traditional Chinese Medicine, Jinan 250355, China; ^2^Bone Biomechanics Engineering Laboratory of Shandong Province, Neck-Shoulder and Lumbocrural Pain Hospital of Shandong First Medical University, Jinan 250062, China; ^3^Shandong First Medical University & Shandong Academy of Medical Sciences, Jinan, Shandong Province, China 250117

## Abstract

**Background:**

Astragalus membranaceus (Huang-qi, AM) and Angelica sinensis (Dang-gui, AS) are common Chinese herbal medicines and have historically been used in spinal cord injury (SCI) therapies. However, the underlying molecular mechanisms of AM&AS remain little understood. The purpose of this research was to explore the bioactive components and the mechanisms of AM&AS in treating SCI according to network pharmacology and the molecular docking approach.

**Methods:**

AM&AS active ingredients were first searched from Traditional Chinese Medicine Systems Pharmacology (TCMSP) and Traditional Chinese Medicine Information Database (TCM-ID). Meanwhile, we collected relevant target genes of SCI through the GeneCards database, OMIM database, PharmGkb database, DurgBank database, and TDD database. By utilizing the STRING database, we constructed a network of protein-protein interactions (PPIs). In addition, we used R and STRING to perform GO and KEGG function enrichment analyses. Subsequently, AutoDock Vina was employed for a molecular docking study on the most active ingredients and most targeted molecules to validate the results of the network pharmacology analysis mentioned above.

**Result:**

The overall number of AM&AS active compounds identified was 22, while the number of SCI-related targets identified was 159. Then, the 4 key active ingredients were MOL000098 quercetin, MOL000422 kaempferol, MOL000354 isorhamnetin, and MOL000392 formononetin. A total of fourteen core targets were TP53, ESR1, MAPK1, MTC, HIF1A, HSP90AA1, FOS, MAPK14, STAT1, AKT1, EGFR, RELA, CCND1, and RB1. The KEGG enrichment analysis results indicated that lipid and atherosclerosis, PI3K-Akt signaling pathway, human cytomegalovirus infection, fluid shear stress, and atherosclerosis, etc., were enhanced with SCI development. Based on the analyses of docked molecules, four main active compounds had high affinity for the key targets.

**Conclusions:**

Altogether, it identified the mechanisms by which AM&AS was used for SCI treatment, namely, active ingredients, targets and signaling pathways. Consequently, further research into AM&AS treating SCI can be conducted on this scientific basis.

## 1. Introduction

Spinal cord injury (SCI) results from damage to the central nervous system caused by various factors, and this disease is one of the major causes of irreversible nerve injury. Depending on the extent of the injury, SCI may result in motor and sensory dysfunction beneath the interface of the injury and the autonomic nerves impaired and bowel, bladder, and sexual dysfunction [1]. Across North America, there are over 1.3 million people who have suffered SCI. The rate of SCI is 30–60 cases per million people [2]. Due to SCI's abrupt onset and high mortality and disability rates, patients experience tremendous mental stress and a significant financial burden [3]. SCI acute phase is marked by pain and sensitivity due to the trauma occurring as well as the concomitant injuries [4, 5]. Currently, the main methods for managing SCI are surgery and nonsurgical treatments, acute phase of SCI conditions are usually treated with opioids and nonsteroidal anti-inflammatories (NSAIDs), and the long-term treatment is however likely to cause serious adverse reactions [6]. Although treatment for SCI has been extensively studied, pharmacological treatment for SCI has not advanced. Thus, research on spinal cord injury has been focused on treatment.

The traditional Chinese medicine (TCM) is also playing crucial role in treating a variety of diseases as a complementary and alternative medicine [7]. Using TCM for SCI treatment can activate the circulation to remove blood stasis and dredging meridian. It is widely known that multiple herbs (namely Astragalus membranaceus (Huang-qi, AM) and the dried root of Astragalus membranaceus (Fisch.)) are used in Chinese herbal formulas, which may produce a large number of metabolites that interact with multiple body targets, thus promoting functional recovery after spinal cord injury [8]. There has been considerable evidence that in addition to its antioxidative, anti-inflammatory, and antitumor effects, AM also has a broad range of pharmacological activities [9]; AM may also reduce apoptosis effects [10]. A recent study found that AM can inhibit the expression of glial fibrillary acidic protein (GFAP) by increasing SOD activity, thereby preventing or reducing secondary SCI. Moreover, high-dose AM injection can reduce the degree of spinal cord edema and improve spinal nerve function with rat spinal cord injury [11]. Angelica sinensis (Dang-gui, AS) is the dried root of Angelica sinensis (Oliv.), a herbal medicine in Asian countries that has been widely used for centuries as a perennial herb. Various pharmacological properties of AS have been documented; among them are immunomodulation, antitumor, antioxidation, anti-inflammation, and neuroprotection [12]. Nevertheless, it is unclear what effect AM&AS has on spinal cord injury, and a deeper understanding of its mechanism and therapeutic effect is needed.

Pharmacology of networks is a cross-discipline based on systems biology and combines systems biology, polypharmacology, computational biology, network analysis, and other disciplines [13]. In addition, numerous researches have demonstrated that network pharmacology is a practical method used to predict drug targets from the perspective of studying TCM macroregulation mechanisms [14]. Hence, we investigated that the potential therapeutic targets and pathways of SCI are treated by AM&AS using network pharmacology, a molecular docking study that was conducted to further predict how AM&AS will recognize and interact with its predicted targets.

## 2. Methods

### 2.1. Construction of Active Ingredient Database and Prediction of Potential Targets of AM&AS

Drug main active ingredients and targets are obtained by using the Traditional Chinese Medicine Systems Pharmacology Database and Analysis Platform (TCMSP, https://tcmsp-e.com/tcmsp.php) and Traditional Chinese Medicine Information Database (TCM-ID, https://ngdc.cncb.ac.cn/databasecommons/). TCM was screened using the oral bioavailability (OB ≥30%) and drug-likeness (DL ≥0.18). PubChem (https://pubchem.ncbi.nlm.nih.gov/) was searched for two-dimensional structures of selected compounds. Compound molecular files were downloaded from PubChem, converted into SDF format, and saved as mol2 files. The target genes were obtained.

### 2.2. Screening for Potential Targets of SCI

We inserted “Spinal cord injury” as keywords. The known therapeutic targets in SCI were also acquired from GeneCards (https://www.genecards.org/), OMIM (https://www.genecards.org/), PharmGkb (https://www.pharmgkb.org/), DurgBank (https://go.drugbank.com/), and TDD (http://db.idrblab.net/ttd/) [15]. Targets associated with drugs and diseases were standardized by UniProt (https://www.uniprot.org/). After retaining the common targets for disease from five database and removing duplicate targets, SCI relevant targets are acquired. By utilizing R package, the AM&AS and SCI targets are drawn in a Venn diagram, and then, the core targets are derived.

### 2.3. PPI Network Analysis and Construction

Common targets for AM&AS and SCI were imported into STRING database (https://cn.string-db.org/) [16]. As long as the species is limited to “Homo sapiens,” the confidence score is greater than 0.90. In Cytoscape (v3.8.0), the PPI file was imported in “TSV” format. For the rest of the parameters, default values were used. The PPI network was obtained visualization.

### 2.4. Constructing Disease-Drug-Ingredient-Target Networks

Genes involved in drug-disease crossover were screened. A number of targets corresponding to AM&AS active ingredients were imported into Cytoscape, as well as predicted targets for SCI disease, and visualization of the network was achieved by creating a network diagram of drug-target-disease interactions.

### 2.5. Analysis of GO and KEGG Functional Enrichment

Core targets were analyzed using GO enrichment analysis and KEGG pathway analysis and the key AM&AS pathway against SCI in order to better understand their functions. A Genome Ontology (GO) knowledgebase (http://www.geneontology.org/) and Kyoto Encyclopedia of Genes and Genomes (KEGG) pathway enrichment analyses (https://www.genome.jp/kegg/) were conducted. Data analysis for GO terms and KEGG pathways was carried out by Cytoscape software and plotted by using the “ggplot” R package. The GO enrichment analysis considers cell components (CC), molecular functions (MF), and biological processes (BP). The results were expressed in the form of a bar graph and bubble maps. Statistical significance was expressed by a *p*-value of <0.05.

### 2.6. Molecular Docking Verifies the Connective Validity of Active Ingredients and Core Targets

By using AutoDock Tool software (version 1.5.6), the connective validity of active ingredients was verified through molecular docking. Structures of ligands used in docking were downloaded from PubChem database; then, all the structures were converted to the mol2 file format. The hydrogen atoms were added to all the ligands and receptor by using AutoDock Tools and conversion structures to PDBQT format. Protein Data Bank (RCSB PDB) (https://www.rcsb.org/) provided crystal structures. After that, PyMOL (Version2.4.0) was run to eliminate small molecules of protein ligands and water molecules, and the PDB format was saved. In the AutoDock Tools, the Lamarckian genetic algorithm was implemented for molecular docking purposes. Using docking free energy as a metric, we organized the docking results. A higher affinity occurs when binding free energies are lower.

## 3. Results

### 3.1. Prediction of Potential Active Ingredients and Chemical Structure of AM&AS

Upon screening of active ingredients, 212 active ingredients were selected between two databases. Based on screening criteria, we filtered out 22 core active components of AM&AS, 20 of which are active ingredients in AM and 2 active ingredients in AS. In accordance with the screening conditions for active ingredients, 192 related key targets were acquired. An overview of information is provided in Table 1.

OB: oral bioavailability; DL: drug-likeness; MW: molecular weight.

### 3.2. Prediction of SCI-Related Targets

A total of 5888 SCI-related targets were obtained through the database of DrugBank, GeneCards, OMIM, PharmGkb and the TDD. 16 related targets were received in the DrugBank, while from GeneCards, 5772 SCI targets were identified. From the OMIM database, 24 SCI-related targets were acquired. According to the PharmGKB database, 69 gene targets related to SCI were identified. Moreover, 7 gene targets were identified from the TDD database. After merger and deduplication of five datasets was performed, 5792 SCI-related targets were identified. As a result of intersecting drug active ingredient and disease targets, 159 targets related to SCI were identified for subsequent analysis. The results are displayed in Figure 1.

### 3.3. Network Construction and Analysis of Protein-Protein Interactions (PPIs)

Protein interactions with the highest confidence (score = 0.9) contain 158 nodes and 208 edges (Figure 2). In the PPI network, proteins are represented by nodes and protein-protein interactions by edges. Small to large values are represented by yellow to red color, respectively.

### 3.4. Building a Network of Drugs, Ingredients, and Target Diseases

Using Cytoscape software, network of drug ingredients, targets, and diseases was built; the results are displayed in Figure 3(a). It is inferred through calculation that there are many interactions between the active ingredient and the key target, so it shows that AM&AS can treat SCI by analyzing synergistic interactions between multiple components, multiple targets, and multiple channels. Hence, Cytoscape's CytoHubba software calculated node degrees, which were used to screen out hub genes. Our screening process excluded seventeen of the main AS&AM ingredients and fourteen of the main targets. Five active ingredients were the following: MOL000098 Quercetin, MOL000422 Kaempferol, MOL000354 Isorhamnetin, and MOL000392 Formononetin. The fourteen core targets were as follows: TP53, ESR1, MAPK1, MTC, HIF1A, HSP90AA1, FOS, MAPK14, STAT1, AKT1, EGFR, RELA, CCND1, and RB1. We used Cytoscape to investigate connections between core targets and thereafter demonstrate the larger node size, indicating that it has a closer relationship with other important targets.  Figure 3(b) illustrates the result.

### 3.5. Enrichment Analysis of GO and KEGG

The GO enrichment analysis was conducted using the R package of the 159 candidate targets and KEGG pathway analysis of these targets for AM&AS treatment of SCI. By GO analysis, a total of 220 GO items, namely, biological processes, molecular functions, and cellular components with *p* < 0.05, were obtained. For each of the top 10 GO items, a bubble chart and a histogram were drawn. There were GO terms associated with response to molecule of bacterial origin and response to metal ion, response to xenobiotic stimulus, response to lipopolysaccharide, etc., in the biological process. Cellular component revealed that coaction targets were mainly enriched in membrane raft, membrane microdomain, postsynaptic membrane, etc. As for molecular functions, targets were mainly related to DNA-binding transcription factor binding, RNA polymerase II-specific DNA-binding transcription factor binding, ubiquitin-like protein ligase binding, etc. (Figures 4(a) and 4(b)).

Further analysis was performed by KEGG pathway analysis on differentially expressed genes to determine which pathways were significantly enriched by these gene changes and elucidated the underlying mechanism of AM&AS-regulated against SCI. As a result of the number of enriched genes, fold changes, and *p* value, Figures 5(a) and 5(b) represent the top 30 pathways. In conclusion, this study indicates that AM&AS exerted that a therapeutic effect for SCI may interact through a number of different signaling pathways, namely, lipid and atherosclerosis, PI3K-Akt signaling pathway, fluid shear stress and atherosclerosis, and human cytomegalovirus infection.

### 3.6. The Docking of Molecules

A list of the top five target proteins (TP53, ESR1, MYC, HIF1A, and MAPK1) of the 14 core active components is selected from the A&S compound-SCI-target interaction network based on their degree over 10. As part of AutoDock's docking process, the active components (quercetin, kaempferol, isorhamnetin, formononetin) are docked molecularly. According to Table 2, the lower docking scores indicate higher binding affinity and stronger receptor-ligand interactions. It is generally the case that the binding energy between ligand and receptor is less than zero, indicating that they can spontaneously bind. As a result of our study, we found that a vast majority of active ingredients and core target proteins had binding energies below −5.0 and showed that active ingredients bind more effectively to core targets. Additionally, these four main active ingredients possess better intermolecular interactions with the protein targets based on our results.

## 4. Discussion

Recent studies have shown that a global increase in socioeconomic and medical costs has been reported for SCI; it is estimated that there are 10.4–83 million cases of SCI annually, and the disease is burdensome to patients and health management organizations [17]. Pathogenesis of SCI involves a primary mechanical injury and multiple secondary injuries induced by subsequent biological processes; among them are apoptosis, local blood flow disorders, hypoxia and ischemia of tissue, infiltration of inflammatory cells, and necrosis of nerve cells [18, 19]. The inflammatory process contributes significantly to damage, so controlling neuroinflammation plays a crucial role in treating SCI [20]. Traditional Chinese medicine is one such drug. Formulas based on TCM always incorporate multiple herbs (multiple components) for a holistic effect described as “multicomponents, multitargets, and multieffects” and played a protective role in the progression of diseases.

Our study used network pharmacologic analysis method to screen the active components of AM&AS. Genes and mechanisms linked to potential pharmacological effects were predicted and elucidated. This resulted in 132 pharmacological targets of AM&AS for SCI treatment, and a total of ten key genes were identified and included TP53, RELA, CTNNB1, MAPK1, and AKT1. Further, our GO and KEGG enrichment analysis demonstrated that AM&AS is effective at treating SCI by regulating inflammation, apoptosis, etc.

A gene functional classification system based on GO annotations is an international standard for gene classification [21]. As a result of GO enrichment analysis, our study inferred the cellular compositions, interface functions, and important biological processes of the core targets. Furthermore, previous research found that pathogenesis of SCI was influenced by inflammatory cytokines and inflammatory response activation [22]. Studies have shown that proinflammatory cytokines, like IL-6, IL-1*β*, IL-17, and TNF-*α*, are integral to the inflammatory response to SCI [23]. Target proteins were significantly enriched in the IL-17 signaling pathway and TNF signaling pathway in the KEGG enrichment analysis, which are closely related to the SCI signal pathway. In addition, PI3K-Akt and p53 signaling pathways were apoptosis-related pathways. It was found that the medicinal components of AM&AS may inhibit the signal pathways such as PI3K/AKT and reduce expression of genes such as AKT1 through mechanisms such as antiapoptosis and reducing inflammation. On the other hand, about KEGG enrichment analysis, the AGE-RAGE signaling pathway is an important signal transduction pathway. Numerous pathogenic processes have been associated with RAGE, namely, cancer, atherosclerosis, inflammatory, and neurodegenerative disease [24]. Therefore, it is therefore essential that the AGE-RAGE signaling pathway be regulated for the development of SCI.

In molecular docking, docking scores are calculated as a result of calculating binding affinity correlations between four main active ingredients and five key targets. Quercetin and TP531 showed the greatest affinity, according to our results (affinity = −7.4 kJ·mol^−1^); additionally, kaempferol and ESR1 showed good binding energy (affinity = −7.3 kJ·mol^−1^). According to these findings, although TP531 and ESR1 are likely to be the primary targets in AM&AS for treating SCI, quercetin and kaempferol could also have potential for treating SCI.

## 5. Conclusions

In summary, from an active ingredient and network pharmacology perspective, this article mainly indicates potential active components and mechanism of AM&AS on SCI treatment. Their possible target genes and related signaling pathways were also preliminarily discussed. However, a simple component-target-pathway analysis may not fully reflect the role of TCM synergistic regulation. Moreover, the research has not yet carried out experimental verification on the key targets and pathways screened by network pharmacology, which is also the limitation of the study. In future work, based on the information provided by network pharmacology, we also plan to explore the key targets and pathways will be further verified at the cellular and animal levels, so as to provide a more sufficient basis for the treatment of SCI with AM&AS.

## Figures and Tables

**Figure 1:** Disease-drug target screening Venn diagram.

**Figure 2:** Network diagram for PPIs.

**Figure 3:** Diagram showing drug ingredients, targets, and diseases. (a) Interaction network of AM&AS compound-SCI-targets. (b) Core target topology.

**Figure 4:** A GO-based functional enrichment analysis. (a) The bubble chart was drawn for the top 10 GO items. Increasing the size of the dot indicates a greater number of genes involved; as the *p* value decreases, the graph becomes redder, and the enrichment increases. (b) A histogram was drawn for the top 10 GO items. A lower *p* value indicates that enrichment is more important; a redder graph indicates a higher enr.

**Figure 5:** KEGG pathway analysis. (a) The top 30 KEGG items were mapped out on the bubble chart. Increasing the size of the dot indicates a greater number of genes involved; as the *p* value decreases, the graph becomes redder, and the enrichment increases. (b) Histogram as drawn for the top 30 KEGG items. A lower *p* value indicates that enrichment is more important; a redder graph indicates a higher enr.

**Table 1:** The main active ingredients in AM&AS.

Herbs	Molecule ID	Molecule name	OB (%)	DL	MW	Molecular structure
Astragalus membranaceus (Huang-qi, AM)	MOL000211	Mairin	55.38	0.78	456.70	
	MOL000239	Jaranol	50.83	0.29	314.29	
	MOL000296	Hederagenin	36.91	0.75	472.70	
	MOL000033	(3S,8S,9S,10R,13R,14S,17R)-10,13-Dimethyl-17-[(2R,5S)-5-propan-2-yloctan-2-yl]-2,3,4,7,8,9,11,12,14,15,16,17-dodecahydro-1H-cyclopenta[a]phenanthren-3-ol	36.23	0.78	428.70	
	MOL000354	Isorhamnetin	49.60	0.31	316.26	
	MOL000371	3,9-Di-O-methylnissolin	53.74	0.48	314.30	
	MOL000374	5′-Hydroxyiso-muronulatol-2′,5′-di-O-glucoside	41.72	0.69	642.67	
	MOL000378	7-O-Methylisomucronulatol	74.69	0.30	316.30	
	MOL000379	9,10-Dimethoxypterocarpan-3-O-*β*-D-glucoside	36.74	0.92	462.49	
	MOL000380	(6aR,11aR)-9,10-Dimethoxy-6a,11a-dihydro-6H-benzofurano[3,2-c]chromen-3-ol	64.26	0.42	300.33	
	MOL000387	Bifendate	31.10	0.67	418.30	
	MOL000392	Formononetin	69.67	0.21	268.26	
	MOL000398	Isoflavanone	109.99	0.3	316.33	
	MOL000417	Calycosin	47.75	0.24	284.26	
	MOL000422	Kaempferol	41.88	0.24	286.24	
	MOL000433	FA	68.96	0.71	441.45	
	MOL000438	(3R)-3-(2-Hydroxy-3,4-dimethoxyphenyl)chroman-7-ol	67.67	0.26	302.35	
	MOL000439	Isomucronulatol-7,2′-di-O-glucosiole	49.28	0.62	464.51	
	MOL000442	1,7-Dihydroxy-3,9-dimethoxy pterocarpene	39.05	0.48	314.31	
	MOL000098	Quercetin	46.43	0.28	302.23	
Angelica sinensis (dang-gui, AS)	MOL000358	Beta-sitosterol	36.91	0.75	414.70	
	MOL000449	Stigmasterol	43.83	0.76	412.70	

**Table 2:** Molecular docking results.

Target	PDB ID	Target structure	Active ingredients	Affinity (kcal·mol^−1^)	Best-docked complex
TP53	6MY0		Quercetin Kaempferol Formononetin Isorhamnetin	−7.4 −6.6 −7.3 −7.2	
ESR1	6KN5		Quercetin Kaempferol Formononetin Isorhamnetin	−7.3 −7.3 −7.0 −7.2	
MYC	1EE4		Quercetin Kaempferol Formononetin Isorhamnetin	−6.6 −7.0 −6.8 −6.9	
HIF1A	3HQU		Quercetin Kaempferol Formononetin Isorhamnetin	−6.8 −6.7 −6.6 −6.7	
MAPK1	6G54		Quercetin Kaempferol Formononetin Isorhamnetin	−7.3 −6.6 −6.5 −6.5	

## Data Availability

The corresponding author can provide data supporting this study upon request.
